The article "Construction and Clinical Application Effect of General Surgery Patient-Oriented Nursing Information Platform Using Cloud Computing" was retracted in 2023. Reasons: signs of a paper mill; suspected computer-generated content; unreliable results or conclusions; concerns about the data.

# Construction and Clinical Application Effect of General Surgery Patient-Oriented Nursing Information Platform Using Cloud Computing

**DOI:** 10.1155/2022/8273701

**Published:** 2022-03-25

**Authors:** Yuanyuan Chen, Jingjing Wang, Weiwei Gao, Dongli Yu, Xiaoxia Shou

**Affiliations:** ^1^General Surgery, Zhejiang Hospital, Hangzhou 310012, China; ^2^Health Management Center, Zhejiang Hospital, Hangzhou 310012, China; ^3^The Nursing Department, Zhejiang Hospital, Hangzhou 310012, China

## Abstract

The paper aims to build a nursing information platform (NIP) for general surgery (GS) patients and explore its clinical application effect based on cloud computing (CC) technology. Specifically, the present work first analyzes and expounds on the characteristics of GS patients, the CC concept, the three-tier service mode of CC, and the cloud data center (CDC). Secondly, based on the principle of the overall system design, the evaluation indexes of medical care end, patient end, family end, and management end are constructed using Visual Studio 2010. Thirdly, the expert evaluation and user evaluation methods are selected to analyze the clinical application effect of the proposed system. Finally, SPSS is used to analyze the effect of the proposed system. The results of the first and second rounds of the expert evaluation show that the authority coefficient of experts is greater than 0.7, which indicates that the degree of expert authority is good. The proposed CC-based GS patient-oriented NIP system is universal. The evaluation results of 20 users have shown 15 doctors and nurses, 14 patients, and 18 family members, who mostly still support applying the proposed CC-based GS patient-oriented NIP system and believe that the system brings convenience and improves work efficiency. In short, more incentives should be taken to build a NIP for GS patients.

## 1. Introduction

With the continuous social development and medical science, people pay even more attention to their Personal Health Care (PHC), especially those patients who may go through such medical treatment as surgery. Generally, complications often occur after General Surgery (GS). Thus, nurses' role as patient care becomes crucial in helping patients recover and providing psychological guidance. To this end, nurses must constantly improve their professional level and nursing service through irregular professional training [1, 2]. As one of the central departments of the hospital, GS is more complex and challenging than other departments in nursing. Therefore, it is imperative to improve the nursing quality and the nursing level of the hospital. Meanwhile, it might substantially help hospitals construct a well-round Hospital Informatization System (HIS) [3, 4].

The article "Construction and Clinical Application Effect of General Surgery Patient-Oriented Nursing Information Platform Using Cloud Computing" was retracted in 2023. Reasons: signs of a paper mill; suspected computer-generated content; unreliable results or conclusions; concerns about the data.

The HIS construction has brought better medical service quality and higher patient satisfaction. At the same time, the hospital is also facing unprecedented challenges [5, 6]. With the continuous expansion of hospital scale and the increasing number of inpatients and outpatients, the business system, together with the construction, relocation, and transformation of various functional buildings, might over-burden the hospital's business system, resulting in higher requirements for the medical secure data storage (SDS) [7, 8]. The resulting problems, such as the continuous expansion of servers, increased space occupation and multiplying energy and labor costs, affect almost all hospitals. In the era of cloud computing (CC) and medical care, the national key planning project is the information construction of the medical industry. There are many types of HISs [9, 10], in which the nursing information platform (NIP) is an integral part of improving hospital clinical efficiency and work quality. Nursing plays a vital role in the actual medical diagnosis and treatment process. Nursing is the leading implementation path of the doctor's prescription and medical advice. Nurses provide direct care for patients to help patients fight against clinal symptoms and ailment-induced psychological problems. Meanwhile, through intimate contact with patients in nursing, nurses can observe and record patients' physiological and psychological situations in real-time [11, 12]. Therefore, establishing a comprehensive NIP will help improve nursing efficiency, reduce nursing errors, and give nurses more time to take care of patients directly [13, 14].

Thereupon, the present work takes medical staff and patients as the main research object and sorts and summarizes the functional modules of the GS patient-oriented NIP based on CC through system tests and functional evaluation methods. Briefly, it analyzes the role of CC in the GS patient-oriented NIP. This research aims to provide some references for constructing a GS patient-oriented NIP.

## 2. Related Theories and Construction Methods of Information Platform

### 2.1. Characteristics of Patients Undergoing GS

After the operation, the patient should be gently escorted to the ward. The medical records of patients with anesthetic surgery should be placed in the corresponding position and updated every time the patient is checked to determine whether the indwelling needle is needed and whether the catheter is smooth [15, 16]. The catheter must be placed appropriately every time, and the sequence must be carried out. The patient must be perfused reasonably. After the surgery, the doctor's instructions and the changes of the patient's vital signs should be closely observed, and the patient's psychological changes must be observed [17, 18]. Meanwhile, nurses must pay attention to patients' various drainage systems and their related properties. Proper routine special care shall be carried out to keep the patient's oral cavity clean and clean the patient's bed in time [19, 20]. After surgery, nurses must always observe the trends and needs of patients, address their needs and then tell the patient and family that the operation is going well. At the same time, the nurse should teach patients postoperative precautions, including posture, diet, and other nursing aspects [21, 22]. (I) Vital signs detection includes measuring the patient's blood pressure according to the size of the operation, the patient's condition, and the doctor's instructions. For patients under general anesthesia, the changes of vital signs should be measured every 15 minutes before waking up and according to the patient's situation. Also, it is necessary to keep the patient's airway stable, pay special attention to the patient's respiratory changes and oxygen saturation, and report to the doctor timely when the patient has sputum and oxygen saturation is less than 95%. (II) Incision and pain care is to observe the patient's incision. If there is excessive bleeding, nurses must report to the doctor in time, find out the cause, and bandage under necessary pressure. Postoperative pain greatly impacts patients' rest, and special attention should be paid to the nature and degree of pain. When the patient is pale and short of breath due to pain, painkillers should be given according to the doctor's instructions, and the effect must be observed. At the same time, medical staff can carry out psychological nursing, distract attention, and reduce patients' pain. (II) The drainage tube and nursing to perfusion: nurses should reasonably arrange the sequence of patients' infusion according to the guidance of doctors to avoid too fast, too rich, and too cold infusion reaction, strengthen the inspection and inform patients of infertility knowledge during perfusion. After the operation, the drainage pipe must be correctly positioned to avoid falling due to blockage and torsion. When the patient gets out of bed, the drainage bag should be placed below the incision to prevent infection caused by retrograde drainage, and the quantity and color of drainage fluid should be accurately recorded. The main psychological characteristics of patients after the operation are as follows: when patients wake up from anesthesia, the success and effect of the operation should be considered immediately. At this time, the nurse should inform the patient of the operation to ensure that the patient remains happy and conducive to recovery.

The article "Construction and Clinical Application Effect of General Surgery Patient-Oriented Nursing Information Platform Using Cloud Computing" was retracted in 2023. Reasons: signs of a paper mill; suspected computer-generated content; unreliable results or conclusions; concerns about the data.

Most patients will feel uneasy after an operation since, no matter the size and duration of the operation, it is a kind of trauma that brings inconvenience to patients, sometimes leading to psychological doubts about the operation's effect. Then, the nurse should first inform the patient that postoperative pain is inevitable and will be relieved and gradually recovered after scientific and reasonable treatment. In exceptional conditions, such as patients with severe mental disorders, there is a need to find out the causes of these disorders and help patients overcome psychological difficulties to receive treatment safely. The nurse must decide the diet duration according to the patient's condition, anesthesia method, and operation position. Usually fasting water for 1-2 days, a liquid diet can be adopted after anal discharge, and the semi-liquid diet can be gradually adopted. Spicy and irritant foods or smoking and drinking are not allowed. After the operation, patients should be advised to eat regularly, eat fewer oranges, and gradually reduce the eating time until the diet is normal. Attention should be paid to help patients maintain a good attitude, work, and rest regularly and interchangeably during this period.

### 2.2. Concept of CC

CC is a new computing model and a service that can provide information technology (IT) resources, applications, and data to users over the network. Today, with the development of IT, CC can bring great changes to the development of small and medium-sized enterprises (SMEs). In particular, CC provides a new service model for delivery and use, through which users can obtain the required services on-demand within the network. The service can be an online application or storage space and other resources. It has the unique advantages of large-scale resource sharing, security, and reliability. The basic idea of CC is to build a giant computer resource pool through network resources and distributed computers, automatically manage and schedule resources, provide services and software-defined user needs, allocate required computing resources, and store each application system (as needed). Therefore, users can devote more energy to their core business without worrying about management details. Meanwhile, CC provides a new way of selling or renting computer resources as commodities to obtain remote application services transmitted through the Internet, thus providing unlimited possibilities and a variety of CC-based services. Lastly, CC itself is traceable and justifiable, and CC service objects can usually be divided into three categories: Software as a Service (SaaS), Platform as a Service (PaaS), and Infrastructure as a Service (Iaas).  Figure 1 shows the three-tier service model of CC.

The article "Construction and Clinical Application Effect of General Surgery Patient-Oriented Nursing Information Platform Using Cloud Computing" was retracted in 2023. Reasons: signs of a paper mill; suspected computer-generated content; unreliable results or conclusions; concerns about the data.

According to the different deployment modes, CC can be a public cloud, private cloud, community cloud, or mixed cloud.  Figure 2 illustrates the analysis diagram of CC elements and characteristics.

Public cloud means that providers provide the public with available resources on the network in payment. Industry Cloud refers to the sharing of resources by multiple institutions with similar needs. The private cloud provides services for an enterprise or company alone. The mixed cloud offers services to different organizations. These four clouds together constitute the CC deployment model.

### 2.3. Cloud Data Center (CDC)

CDC is developed from the traditional data center based on CC technology. The computer room infrastructure is more or less the same as the traditional data center, only with larger scale, higher integration, and much-improved service levels. CDC hosts computing, storage, and other resources, manages and safeguards the backbone infrastructure platform uniformly, transmits data through the network, and provides users with available computing services. The solutions of the background CDC and the whole IT department complement each other, uniformly manage and maintain the software and hardware, and continuously debug the CC platform at the software level according to the actual business load. In contrast, the hardware level ensures the normal operation of the CC platform and the allocation of computing, storage, network, and other resources to ensure the computer room's normal environment. Users can have enough computing or storage resources without worrying about the background, just like household water and electricity usage.

The main features of CDC are as follows: (I) It uses virtualization technology (VT) to manage abstract resources, eliminates heterogeneous systems barriers, and quickly deploys resources and services. (II) It realizes the unified deployment of computing, storage, and network resources through automation and intelligence and provides enterprise-oriented resource customization services. CC platform resources are abstracted and isolated from each other, which solves the compatibility problem between application platforms. (III) It combines VT and green technology and intelligent and efficient energy management and environmental control system, reduces Energy Consumption (EC), and realizes green data. To sum up, CDC has the advantages of high resource utilization, convenient management and maintenance, lower investment costs, highly-compatible with different resource platforms, and smooth transfer of activities. Lastly, the CDC application will fill the gap of the traditional data center.  Figure 3 demonstrates the main features of CDC.

The article "Construction and Clinical Application Effect of General Surgery Patient-Oriented Nursing Information Platform Using Cloud Computing" was retracted in 2023. Reasons: signs of a paper mill; suspected computer-generated content; unreliable results or conclusions; concerns about the data.

### 2.4. Implementation of Medical Cloud Desktop Solution

According to the analysis of the current situation of the hospital, managing many computer terminals scientifically and efficiently is the most urgent problem in hospital information management. To this end, this section proposes a frugal cloud desktop virtual office based on infrastructure. All office environments and other medical workstations, reservation, and invoice windows work in the cloud of CDC and provide the service form of virtual user environment. Specially, all the user's desktops are deployed on the CC platform, requiring little maintenance. As long as the terminal browser can access its desktop environment, it adopts virtual desktop infrastructure. The CDC completely controls the cloud office environment to realize centralized management, centralized deployment, centralized security protection, and remote maintenance. Cloud space is independent of each other, and each user has its own data space. Users can configure a custom desktop. Medical data are stored in the CDC to ensure data security. The cloud office also complements the CDC application and maximizes resource utilization and management. Meanwhile, it relies on the background cloud infrastructure to provide strong technical support through servers, storage, and network resources. Cloud desktop terminals are usually thin clients, such as processors, memory, and flash memory without hard disks and fan design. They can also be terminal devices, such as computers, smartphones, and tablets.

At present, desktop VT is relatively mature technically supported by many cloud service providers. Cloud services can be easily deployed through desktop virtualization software based on the robust CDC infrastructure, which is relatively easy for each hospital to accept and deploy. Virtual office infrastructure technology provides office distribution systems by providing rapid response-ability, personalized user experience, centralized management, overall office system image, utilization advantage and maintenance management, and security provided by CDC. The design architecture of the cloud desktop is shown in Figure 4. Cloud desktop has five characteristics: first, it gives users an incredible experience, namely, barrier-free printing. Second, a virtual desktop can be used to manage, schedule, and deploy the whole cloud desktop system. Third, the applications can be deployed more rapidly, and the application transference can be simplified through VT. Fourth, the mature link cloning technology can use the template method to create multiple virtual desktops quickly. Fifth, the CC background is a cloud infrastructure service platform and is built through VT.

The article "Construction and Clinical Application Effect of General Surgery Patient-Oriented Nursing Information Platform Using Cloud Computing" was retracted in 2023. Reasons: signs of a paper mill; suspected computer-generated content; unreliable results or conclusions; concerns about the data.

## 3. Design of NIP and Questionnaire Survey (QS)

### 3.1. Design of NIP

The NIP design includes overall design, modular design, database design, CC-based GS patient-oriented NIP design, coded by the object-oriented language, software engineering theory, and CC technology. The present work adopts the Visual Studio 2010 development tool to realize each system function from the user's needs based on some general principles, including advanced and practical principles, normative principles, openness principles, openness principles, and quick response principles.

Modular design is to design corresponding subfunction modules according to user requirements.  Figure 5 specifies the business flow chart.

The database design includes data integrity design, database logic design, and database logic structure design. According to the entities involved in the GS patient-oriented NIP, Figure 6 designs the entity-relationship diagram.

The subsequent research selects appropriate test environments and indexes and uses the classical V model to test the proposed GS patient-oriented NIP. The whole test process is carried out gradually from left to right.  Figure 7 depicts the schematic diagram of the classic V model.

### 3.2. QS Design

This section systematically has scored experts, nurses, and patients in a hospital to develop a NIP system to meet the user needs. There are two rounds of expert index evaluation, including evaluating medical care end, patient end, family end, and administrator end. Importantly, the QS has gained the hospital and patients' consent, and their anonymity and confidentiality will be guaranteed. Informed consent has been signed. A total of 20 patients are interviewed, with a recovery efficiency of 100%. The reliability and validity of the collected QS are analyzed by SPSS, finding that the designed QS has good reliability and validity. Several key points involved in the QS are listed in Table 1.

## 4. Test Results and QS

### 4.1. Test Result

The proposed CC-based GS patient-oriented NIP adopts very mature development technology.  Table 2 unfolds the test results of the proposed NIP system.

The proposed GS patient-oriented NIP performance test results are enumerated in Table 3.

Tables 2 and 3 imply that the proposed CC-based GS patient-oriented NIP test results are good and can meet the needs of nurses and patients.

### 4.2. Coordination Degree of Expert Opinions

First, Figure 8 analyzes the coordination degree of expert opinions.

The article "Construction and Clinical Application Effect of General Surgery Patient-Oriented Nursing Information Platform Using Cloud Computing" was retracted in 2023. Reasons: signs of a paper mill; suspected computer-generated content; unreliable results or conclusions; concerns about the data.

Figure 8 analyzes the coordination degree of expert opinions at the medical care end, patient end, family member end, and management end of the index. *W* is taken between 0 and 1. The greater *W* is, the better the coordination degree is. Apparently, the coordination degree of experts from the first round to the second round is also getting higher.

### 4.3. Expert Consultation Results

Figure 9 display the expert consultation results to evaluate the importance and feasibility of the proposed NIP.  Figure 10 describe the results of the first round and second round of expert consultation, respectively.

In general, when the expert authority coefficient is greater than 0.7, the expert's authority degree is better. The higher the expert authority coefficient, the more reliable the result is. Figures 9 and 10 suggest that the first and second round expert authority coefficients are 0.84 and 0.85, respectively. Thus, experts have a high degree of authority.

### 4.4. User Attitude

Figure 11 examines the hospital and patients' attitudes towards the proposed NIP.

Figure 11 corroborates that most medical staff, patients, and family members support using the proposed NIP. The willingness to use the system can be obtained from the QS results. Specifically, there are 15 medical staff, 14 patients, and 18 families in total. Members who are hesitant to use the system include three doctors and nurses, four patients, and one family member. Two doctors, two patients, and one family member are unwilling to use the proposed NIP. The main reason is that they are worried about the system's stability, such as the system response and convenience. Moreover, how well nurses can operate the proposed system should be fully considered in the design process and practice of the system. To sum up, most of them still support applying the proposed NIP system in surgical nursing and believe that the proposed system brings convenience and improves work efficiency.

## 5. Conclusion

Based on the technologies related to CC and system design, the present work analyzes the characteristics of GS patient-oriented surgical nursing and puts forward the relevant definitions of surgical nursing. Then, relying on the methods of system test and function test, the present work analyzes the effect of the system in clinical application and briefly explores the relationship between the system functional modules based on the overall design principle of the system. Finally, it constructs the GS patient-oriented NIP system based on CC. The results show that the authority coefficient of experts is greater than 0.7, which shows that the degree of expert authority is good, and the proposed system is universal. The evaluation results of 20 users have shown that there are 15 doctors and nurses, 14 patients, and 18 family members. They mainly worry about the system's stability, response time, convenience, and nurse-operability. Overall, most of them still support applying the system in surgical nursing and believe that the proposed system brings convenience and improves work efficiency. In a word, the construction of GS patient-oriented NIP can promote the development of medical work.

The article "Construction and Clinical Application Effect of General Surgery Patient-Oriented Nursing Information Platform Using Cloud Computing" was retracted in 2023. Reasons: signs of a paper mill; suspected computer-generated content; unreliable results or conclusions; concerns about the data.

The present work constructs a GS patient-oriented NIP based on CC technology. Affected by the actual experimental conditions, the selected research samples are limited and not enough to cover the whole. The samples will continue to be expanded and analyzed in the later research. Meanwhile, only the single function of functional modules is considered in the system design process. Given the theme of the article, there is no in-depth discussion. More factors will be considered in the follow-up research.

## Figures and Tables

**Figure 1:** CC three-tier service model.

**Figure 2:** Analysis of CC's elements and characteristics.

**Figure 3:** Main features of CDC.

**Figure 4:** Logical architecture diagram of cloud desktop.

**Figure 5:** System business flowchart.

**Figure 6:** System entity relationship diagram.

**Figure 7:** Classical V model.

**Figure 8:** Expert coordination degree.

**Figure 9:** The first-round expert evaluation results on indexes.

**Figure 10:** The second-round expert evaluation results on indexes.

**Figure 11:** User attitudes.

**Table 1:** Key settings of the QS.

Index	Index content	Feasibility					Importance				
Medical end	Nurse login, nurse information management, doctor's order copying, doctor's order checking, doctor's order execution, patient query, event report, and quality standard	5	4	3	2	1	5	4	3	2	1
Patient end	Patient information exchange, view doctor's orders, event reports, and view relevant health knowledge	5	4	3	2	1	5	4	3	2	1
Family end	Participate in the management of patients' surgical nursing services	5	4	3	2	1	5	4	3	2	1
Administrator side	Manage and maintain the platform	5	4	3	2	1	5	4	3	2	1

**Table 2:** Test results of the proposed NIP system.

Test scenario number	Operation function	Expected output	Test result
PC&MP-1	Nurse login	Enter the account and password and log in to the system	Pass
PC&MP-2	Nurse information management	Fill in and modify your personal information	Pass
PC&MP-3	Doctor's order copying, doctor's order checking, doctor's order execution	Enter the corresponding page for the corresponding operation	Pass
PC&MP-4	Patient inquiry	Enter the patient query interface, enter the patient number and query the patient information and status	Pass
PC&MP-5	Event report	Open the event report page, fill in the event information and click report	Pass
PC&MP-6	Quality standard	Enter the page, modify the quality standard and click submit	Pass

The article "Construction and Clinical Application Effect of General Surgery Patient-Oriented Nursing Information Platform Using Cloud Computing" was retracted in 2023. Reasons: signs of a paper mill; suspected computer-generated content; unreliable results or conclusions; concerns about the data.

**Table 3:** Performance test results of the proposed NIP.

Test scenario number	Operation function	Scene description	Average corresponding time (s)	Test result
PC&MP-7	Nurse login	One user every two seconds, and then run for 15 minutes	0.062	Pass
PC&MP-8	Nurse information management	One user every two seconds, and then run for 15 minutes	0.171	Pass
PC&MP-9	Doctor's order copying, doctor's order checking, doctor's order execution	One user every two seconds, and then run for 15 minutes	0.156	Pass
PC&MP-10	Patient inquiry	One user every two seconds, and then run for 15 minutes	0.161	Pass
PC&MP-11	Event report	One user every two seconds, and then run for 15 minutes	0.108	Pass
PC&MP-12	Quality standard	One user every two seconds, and then run for 15 minutes	0.153	Pass

## Data Availability

The simulation experiment data used to support the findings of this study are available from the corresponding author upon request.
